# Innovation and Reform of Ideological and Political Course Mode in Colleges and Universities Based on Big Data Network Platform

**DOI:** 10.1155/2022/1036168

**Published:** 2022-09-16

**Authors:** Dandan Qiu

**Affiliations:** College of Marxism, Jilin Jianzhu University, Changchun, Jilin 130008, China

## Abstract

With the continuous development of the computer field, the Internet has become the main way of education in today's era. The development of computer technology and big data has brought innovation and opportunities to the teaching mode of ideological and political courses in colleges and universities. Due to the dynamic change of big data, there are many difficulties in the establishment of ideological and political course models in colleges and universities. This paper studies the innovation of ideological and political course modes in colleges and universities on the network platform under the background of big data. This paper mainly compares the traditional teaching mode and explores the formal modeling method of network platform education. The discrete dynamic modeling technology of the complex system is used to model the formal process of online education. Then, it carries out nonlinear prediction modeling for the operation efficiency and traffic change of the network platform under the big data environment and uses dynamic modeling to predict the learning effect of college students' ideological and political course mode. The results show that the formal method of education under dynamic modeling can improve the defects of traditional teaching and give full play to the advantages of network platform teaching. Improving the teaching mode of network platform can improve students' learning efficiency. Finally, in the dynamic model prediction, the problem of big data affecting the model results is improved, and the accuracy of the prediction model is improved.

## 1. Introduction

According to the statistics of network information platforms, the student group accounts for the largest proportion in the classification of Internet users [1] followed by workers and journalists. Most students have mastered the basic user functions of the Internet and can independently query, obtain information, and communicate [2]. Therefore, the teaching environment in colleges and universities should also be optimized and improved in combination with network technology [3]. Combining the traditional teaching mode and educational concept with new technology to adapt to the development of the times is our focus [4]. The main work of ideological and political courses in colleges and universities is to establish the correct three concepts and improve students' moral quality and political level. The ideological and political theory course undertakes the task of systematic Marxist theory education for college students. It is an important position to consolidate the guiding position of Marxism in the ideological field of colleges and universities and adhere to the direction of socialist school running. It is the main channel and core course to comprehensively implement the party's educational policy and the fundamental task of building morality and cultivating people. It is the soul course to strengthen and improve the ideological and political work in colleges and universities and realize the connotative development of higher education. With the promulgation of national policies, many schools have focused on the content of ideological and political education [5]. However, the traditional teaching mode and concept are relatively single and cannot be better integrated into Internet thought [6]. Due to the limitations of technical means and analysis methods, the collection of students' various demands and information mainly adopt the form of a manual sampling survey, but this form will make the survey results too general and inaccurate. Using inaccurate information as the basis for carrying out ideological and political theory teaching activities in colleges and universities will obviously directly affect the effectiveness of education. With the introduction of information technology, many schools gradually began to adopt online teaching mode and integrate Internet information to carry out education. With the use of the network platform, the teaching content of ideological and political courses in colleges and universities has been gradually enriched and the teaching environment has been improved [7]. The network platform model under the big data environment cannot only open the school's publicity channels, reduce the school's education cost but also expand the scope of students' communication [8, 9]. Because online education is different from the traditional education model, although it can improve students' participation in the classroom, there are also problems such as face-to-face communication between teachers and students [10]. Based on the abovementioned situation, many educational researchers have proposed to apply big data dynamic modeling technology to college classroom models. Dynamic modeling is a technology for processing dynamic data supported by complex systems [11]. It can filter interference data in massive data information and get accurate results. At present, the formal teaching modeling proposed by combining big data technology with subject theory teaching is the main method to deal with the defects of network platform teaching mode [12]. At present, China's Internet coverage is gradually expanding, and mobile terminals are widely popularized. On the basis of continuing to adhere to the traditional advantages, the ideological and political theory course in colleges and universities should actively realize the integration, mutual assistance, and progress with big data technology, form a new idea of combining traditional advantages with big data technology, and enhance the liveliness and attractiveness of the traditional model. For example, we can use the support of big data information and network technology to conduct preclass research and prediction; in class monitoring and analysis; and after class inspection and feedback are integrated into the whole process of lesson preparation, teaching, and assessment of ideological and political theory courses.

This paper is mainly divided into three parts. The first part briefly describes the main problems and solutions of the network platform mode of ideological and political courses in colleges and universities under the big data environment and analyzes the application status of dynamic modeling technology in various countries. The second part mainly uses big data dynamic modeling technology to study the formal modeling of ideological and political course modes. Finally, it explores the operation efficiency and influencing factors of network platforms under the background of dynamic data, and forecasts the learning effect of students' network platforms through the prediction model of complex systems. The third part analyzes the results of the research on the dynamic modeling of the network platform in the mode of ideological and political courses in colleges and universities under the background of big data.

## 2. The Related Works

With the advent of the big data era, many schools use computer technology to form a dynamic interactive platform to carry out educational work [13]. Most online education platforms can change the complex process in the traditional teaching mode and simplify students' learning process [14]. The dynamic information of the Internet is used as the current news in the learning content, and the teaching demonstration is carried out by means of video, audio, pictures, and so on. The traditional teaching mode has some problems, such as the teaching content is not direct, while the online environment of the network platform can intuitively show the students' learning content and let the learners form a three-dimensional knowledge impression [15]. However, in the Internet big data environment, students will encounter a lot of bad information when using the network platform. This bad information and useless news will have a bad impact on students' physical and mental content [16]. The emergence of a lot of junk information is easy to make immature, unstable three values and poor judgment students have confused cognition [17]. There are no strict regulations on the use of network platforms. This loose network environment is easy for students to express their own comments and opinions. If students' moral quality is affected, it will have an irreparable impact [18]. Therefore, with the support of big data information, we need to build an ideological and political course network platform education model to improve students' learning environment. In the construction of ideological and political network platform, we should pay attention to updating the concept of ideological and political education; expanding the space and channels of ideological and political education by using modern and advanced network information means; improving the pertinence, effectiveness, attractiveness, and appeal of ideological and political education; actively exploring effective ways to innovate the ideological and political education of college students; and gradually forming a theme website target orientation that conforms to the ideological reality of our students. Let students combine ideology and morality with the use of the Internet. In order to distinguish between bad information and interference data, we use dynamic modeling technology to formally model the teaching mode [19].

The UK combines big data dynamic modeling technology with information network structure to form an intelligent information processing system [20]. Research on multi-source data fusion in complex data information environment. The combined dynamic modeling technology is applied to the power system to solve the problems of poor data test accuracy in power engineering.

The United States focuses on the privacy of Internet information, and they are ahead in the development of big data technology [21]. With the rapid efficiency of data flow, security and privacy have become the focus of people's attention. In order to solve the problem of poor performance of privacy protection systems, researchers proposed the modeling of complex network security systems. The experimental results show that the security system can effectively protect users' personal information.

French researchers applied dynamic modeling technology to severe weather prediction [22]. With the expansion of global warming trend, bad environment and bad weather occur frequently. Many cities are vulnerable to tornadoes and rainstorms. The establishment of risk early warning and prediction models based on big data complex systems can improve people's ability to judge the environment. This model cannot only predict environmental changes but also carry out a risk assessment and loss assessment [23, 24].

China applies big data dynamic modeling technology to the field of education, including data modeling in mathematics classrooms [25, 26]. Let students intuitively understand the changes and principles of mathematical models. With the continuous improvement of people's living standards through big data technology, ideological, and political education is also an open and complex system. Based on the development status of big data dynamic modeling technology in various countries, this paper puts forward the research on dynamic modeling in the network platform mode of ideological and political courses in colleges and universities under the big data environment.

## 3. Research on Dynamic Modeling of Ideological and Political Course Mode Innovation in Colleges and Universities Based on Big Data Network Platform

### 3.1. Research on Formal Dynamic Modeling of Ideological and Political Education in Colleges and Universities Based on Big Data Network Platform

At present, Internet online platform teaching has become the main research direction of the new education model. Compared with the traditional teaching environment, online teaching has many defects, which cannot meet the requirements of face-to-face communication between teachers and students. The interactivity is poor because the teaching process does not require strict synchronization in time and space, resulting in poor interactivity. Students cannot put forward the problems encountered in the process in a timely and effective manner, nor can they give clear and clear answers in real-time. Although the technology of enhancing interactivity is widely used in the teaching process, its effect is much inferior to that of traditional process communication, which is also a disadvantage. In order to overcome the defects of network platform teaching mode, we need to integrate big data technology and education methods. In the process of ideological and political teaching in colleges and universities, teaching activities are an auxiliary coordination way. In order to intuitively analyze the teaching process of ideological and political courses and effectively guide students' learning activities, we need to practice educational principles. The analysis teaching process is divided into two stages. One is to analyze the learning content, the other is to analyze the teaching process. Only under the condition of mutual adaptation and integration can a correct teaching method be formed. The teaching process of ideological and political courses mainly includes lesson preparation, lecture, homework after class, homework correction, and so on. The learning process is divided into preview, listening, review, and other stages. In order to explore the innovative content of ideological and political course models in colleges and universities, we need to analyze the relationship between professors and learners, as shown in Figure 1.

It can be seen from Figure 1 that the teaching link and learning link are connected and adapt to each other. They interact and can influence each other. The first stage is the key premise of imparting knowledge, and the second stage is the core content of the teaching process. Through the analysis of the relationship between them, we can know that the teaching mode of ideological and political courses is not only a complex system structure but also a nonprocess and nonlinear link. Network platform system is also a computer system, which needs to be formalized strictly. Therefore, we formally model the teaching mode of ideological and political courses in colleges and universities and build a network platform for ideological and political course teaching systems. This formal modeling is dynamic. Through the analysis of asynchrony in the learning process, we know that teaching and learning are interrelated. In addition, the educational process also includes concurrency and uncertainty. The comparison of the distribution of online education on the network platform shows that the traditional teaching mode cannot share resource information. In dealing with this sharing mode, we use discrete dynamic modeling Petri net to analyze it. Petri net is a tool for describing data in large data complex systems. It can effectively deal with concurrent, distributed, and uncertain data information. In the data system, we will use Petri nets to analyze the stability of the system before and after processing big data, as shown in Figure 2.

It can be seen from Figure 2 that with the increase in the amount of data to be processed, the modeling system optimized by Petri net can quickly solve complex data problems and improve the stability of the model. Compared with the traditional system without Petri net optimization, its functionality has been effectively improved. System variables need to be initialized and defined first as:

(1) $$\begin{array}{c} N_{1}=B;E;F;c_{in}\text{.} \end{array}$$

After the initialization definition, we define the modality of the directed variables of the basic network as:

(2) $$\begin{array}{c} c_{in}=\left\{s_{1},s_{2},s_{3}\right\}B=\left\{s_{1},s_{2},s_{3},s_{4}\right\}E=\left\{a,b\right\}\text{,} \end{array}$$

where *B*={*s*_1_, *s*_2_, *s*_3_, *s*_4_} is the condition set and *E*={*a*, *b*} is the event set. The whole system is a completely closed structure with connectivity. After the condition content and event content are specially defined, we can simulate the data information of the initial system. When the difficulty of learning content is different, we find that a formal system can be used for teaching description. Because there are many definitions of elements in the teaching link, most of them have their own meanings, so we need to add Petri nets for formal descriptions. Firstly, the elements generated in teaching activities are classified, and then the formal dynamic modeling model of ideological and political course network teaching under Petri net system is constructed, as shown in Figure 3.

As can be seen from Figure 3, the nodes of the system structure include variable parameters, which are mainly composed of teacher status, student status, teaching materials, teaching purpose, etc. According to the formal dynamic modeling model, we can define the modeling formula of the system as:

(3) $$\begin{array}{c} \psi =R,T,F,C,I_{-},I_{+},M_{0}\text{.} \end{array}$$

The abovementioned variables are the meanings of nodes in the corresponding system. Due to the teacher's class process, students can ask questions and answer questions independently. Therefore, Petri net is a simplified system of adaptive cyclic rules. It can eliminate the unnecessary process in the teaching link and improve the operation efficiency of the whole model. Compare the operation efficiency of the network platform teaching system before and after Petri net optimization, as shown in Figure 4.

It can be seen from Figure 4 that the teaching system optimized by dynamic modeling Petri net can process a large amount of student information. With the increase of student data, the operation efficiency of the system does not decline. The course of dynamic data modeling includes theory and practice. For the theoretical course of ideological and political courses, we mainly use the modeling method to improve it. Be able to analyze students as the main body of learning. Firstly, take examples as cases in the network platform, and take mastering knowledge and learning ideas as the key content of cultivating students. According to the complex information in the big data environment as the basis for knowledge expansion, students will be brought into the actual problem situation for learning. Finally, for the purpose of correctly expressing their ideas, the learning effect is displayed in the form of dynamic modeling. According to the abovementioned research, Petri net can optimize the performance of the whole network teaching platform and provide effective technical support for the innovation of ideological and political course modes in colleges and universities.

### 3.2. Research on Dynamic Modeling of Learning Effect Prediction of College Ideological and Political Course Network Platform Based on Big Data Environment

Compared with the traditional teaching mode, teachers on the network teaching platform cannot accurately grasp the current learning state of students. Through the investigation, it is found that most students' learning attitude in the online teaching process is not correct, and their class concentration is not strong. They are often late for the first online class in the morning, and they cannot answer the questions by roll call in class. Some students even use their computers to have classes while playing games on their mobile phones. Some students even sleep while listening to the online live class. According to the background data of superstars, the ratios of submitting homework and completing homework are 46% and 65%, respectively. Students often ask their teachers to hand in their homework after class. With the popularization of network teaching platforms, the resource information of related courses is becoming more and more extensive. Online teaching has become an indispensable member of the classroom of primary and secondary schools. In the big data environment, when the network platform uses teaching resources, it is easy to produce a large number of garbage data and browsing records. Some of these browsing records can represent students' learning traces and learning status. Through the analysis and retrieval of historical trace information, we can immediately understand the learning effect of students on the network platform. Before the prediction of students' learning effect, it is necessary to analyze the data flow in the big data system and detect the length and efficiency of students' learning according to the change in data flow. Big data dynamic modeling technology can model and predict the data flow and judge the changing trend and historical trend of the whole network data. Then the prediction results are provided to teaching workers to analyze the use effect of the platform independently. In the use of prediction models, most researchers use periodic modeling to predict and analyze the trend according to the periodic changes in data. However, periodic modeling can only describe the local change characteristics of data flow, not the change of dynamic data. The stability of periodic model is also poor, and the accuracy of model prediction decreases with the increase of users. Therefore, this paper uses big data dynamic discrete modeling to improve the prediction effect of the system. We use the computing model to process massive data, form a distributed state, and define the discrete model. The basic working principle is to divide the data into small sets of tasks and use different nodes to execute the tasks. In order to solve the bottleneck problem of the model, we define input variables, storage variables, and output variables as:

(4) $$\begin{array}{c} u\left(n\right)={\left(u_{1}\left(n\right),u_{2}\left(n\right),\ldots ,u_{K}\left(n\right)\right)}^{T}\text{,}\\ x\left(n\right)={\left(x_{1}\left(n\right),x_{2}\left(n\right),\ldots ,x_{N}\left(n\right)\right)}^{T}\text{,}\\ y\left(n\right)={\left(y_{1}\left(n\right),y_{2}\left(n\right),\ldots ,y_{L}\left(n\right)\right)}^{T}\text{,} \end{array}$$

*u*(*n*), *x*(*n*), and *y*(*n*) are input, storage, and output variables, respectively. At a certain time, the updated state equation and calculation formula of the network system are as follows:

(5) $$\begin{array}{c} x\left(n+1\right)=f_{1}\left(W^{in}u\left(n+1\right)+Wx\left(n\right)\right),\\ y\left(n+1\right)f_{2}\left(W^{out}u\left(n+1\right)\right)\text{.} \end{array}$$

In the formula, *W*^in^, *W*^out^, *f*_1_, and *f*_2_ represent the parameter connection weight value and activation function of the computer system, respectively. The steps of the whole system structure are as follows: initialize according to the problem, define parameter variables, and establish the expected relationship between parameter samples and prediction samples. In the feedback elimination state, the abovementioned variable parameters are fixed, and the following formula can be obtained by training the subsequent model as:

(6) $$\begin{array}{c} W^{out}x\left(n\right)\approx y_{t}\left(n+1\right)\text{.} \end{array}$$

According to the formula, it can be judged that the vector *x*(*n*) is represented by *u*(*n*), and the relationship between them is:

(7) $$\begin{array}{c} u\left(n\right)⟶y_{t}\left(n\right)\text{.} \end{array}$$

We represent the state vector of the participation matrix with the training objective:

(8) $$\begin{array}{c} Y=W^{out}X\min\;{\left|Y-Y_{t}\right|}^{2}W^{out}=Y_{t}\times X^{+}\text{.} \end{array}$$

There is an inverse matrix definition in the abovementioned formula and the variable *X*^+^ is the parameter representative of the inverse matrix. Finally, the actual output value is predicted according to the training results as:

(9) $$\begin{array}{c} \hat{y}\left(n\right)=W^{out}x\left(n\right)\text{.} \end{array}$$

We compare the big data dynamic modeling technology with the traditional modeling technology to explore their operation speed in processing a large amount of data, as shown in Figure 5.

It can be seen from Figure 5 that the big data dynamic modeling technology can handle the calculation of dynamic complex data and improve the running speed of the model. The traditional modeling technology image is a falling curve, and the operation will be slower with the increase in the amount of data. Finally, according to the changing trend of big data information, this paper analyzes the learning effect of students' ideological and political courses on the online platform. In this paper, the decision tree algorithm ID3 in discrete dynamic modeling is used for research. This algorithm has high calculation accuracy and dynamic data processing function. ID3 algorithm takes the data as the variable of node redundancy and uses node splitting for evaluation. The node definition formula is as follows:

(10) $$\begin{array}{c} Entropy\left(t\right)=-\overset{c}{\underset{c=1}{\sum }}p\left(\left.c\right|t\right)\log_{2}\;p\left(\left.c\right|t\right)\text{.} \end{array}$$

In practice, in order to avoid the over-fitting problem of data, we usually use the data growth rate instead of the evaluation standard. We randomly selected the academic performance of some students in the university database as the prediction data. First, compare the performance trends of students in various subjects, as shown in Figure 6.

As can be seen from Figure 6, there is little difference between the average score for Chinese and ideological and political courses, and the score for mathematics is poor. In contrast to the above, in order to test the effectiveness of the model, we divide the students into two parts. One part adopts the traditional offline teaching mode; the other part adopts the network platform teaching mode. A control group was established to track the ideological and political and Chinese scores of the students in the two parts, as shown in Figure 7.

It can be seen from Figure 7 that the scores of students, who use the network platform to teach ideological and political courses and Chinese courses have been improved, and the rising effect of ideological and political courses is greater than that of Chinese courses. Therefore, it can be proved that the high-efficiency ideological and political course model innovation system based on a big data network platform has a positive impact on students' learning effect. The traditional ideological and political education is mainly based on the simple indoctrination education mode, which is boring and lacks of vividness and flexibility. Network ideological and political education takes advantage of the characteristics of a large amount of network information, fast transmission speed, and strong influence, integrate other media, such as newspapers, radio, and television, enriches the content of ideological and political education, so as to enhance the attraction of network ideological and political education, and also enable the educated students to receive information independently and sublimate their thoughts.

## 4. Analysis of Dynamic Modeling Research Results of Ideological and Political Course Mode Innovation in Colleges and Universities Based on Big Data Network Platform

### 4.1. Analysis of Research Results of Formal Dynamic Modeling of Ideological and Political Education in Colleges and Universities Based on Big Data Network Platform

In the process of school education, the level of students' learning ability is not balanced. We divide students' learning ability into low level, intermediate level, and high level. In order to study the impact of big data network platforms on the innovation of ideological and political course modes in colleges and universities, we analyze the characteristics of teaching activities in the school and require teachers to teach only one specified course at the same time. Set the learning process of students as preview and review, and judge the learning situation of students at three levels according to the length of learning time. Students' basic learning knowledge shall be evaluated according to the content of the syllabus, as shown in Figure 8.

It can be seen from Figure 8 that students with advanced learning abilities have the best performance in learning on the network platform. With the increase in review and preview time, the performance changes more and more. Therefore, we can judge that students with low learning ability can improve learning efficiency after preview and review. Therefore, the system optimized by Petri net can achieve positive help to students' achievement in dealing with nonlinear formal teaching.

### 4.2. Dynamic Modeling and Analysis of Learning Effect Prediction of College Ideological and Political Course Network Platform Based on Big Data Environment

To explore the nonlinear prediction principle of data flow in the big data environment, we first need to collect a certain range of data history traces. Finally, the historical traces are divided to obtain multiple subset training samples. Finally, discrete dynamic modeling technology is used to predict the sample data. In database selection, we set one server as the initial node and the other three as auxiliary nodes. In order to analyze the advantages of data modeling, we compare the accuracy coefficient of experimental results between traditional modeling algorithm and big data dynamic modeling algorithm, as shown in Figure 9.

As can be seen from Figure 9, the accuracy of traditional modeling technology is significantly reduced by increasing the amount of data. The accuracy of the dynamic modeling technology studied in this paper remains above the standard coefficient. Therefore, dynamic modeling technology is effective and applicable to the performance of prediction models. In exploring the impact of network platforms on ideological and political courses in colleges and universities, we mainly analyze the learning effect of students. With the increase of the characteristic coefficients of the decision tree model samples, the training time of the model becomes longer. The more complex the structure of the model, the higher the degree of calculation, resulting in poor applicability and feedback efficiency of the model. We divide students' midterm test scores, ordinary quiz scores, and final exam scores into data of the same level. In order to improve the efficiency and accuracy of the prediction model, we use the cross-validation method to test. The data are randomly divided into several parts, half of the set is selected as the training data, and the other part is the control data. There are many influencing factors in the learning effect of students' network platforms, among which the effect of after-school homework is the greatest. We compared the time of students' online classes with the prediction rate of achievement change. Explore the gap between the predicted effect and the actual effect, as shown in Figure 10.

As can be seen from Figure 10, with the increase in students' class time on the network platform, the scores show a positive curve change. There is little difference between the prediction coefficient of dynamic data modeling and the actual coefficient, so the dynamic data modeling technology in the big data environment can accurately analyze the influencing factors and change trend of the network platform on students' learning effect.

## 5. Conclusion

With the Internet big data environment gradually improving people's lifestyles, school education has also established a new model. Most schools have adopted the network platform for teaching. Different from traditional teaching methods, students and teachers cannot communicate face-to-face. Therefore, teachers cannot accurately grasp students' feedback to the classroom, nor can they grasp students' current learning state. Based on the abovementioned situation, this paper studies the innovation of ideological and political course modes in colleges and universities on the big data network platform. Firstly, the big data dynamic modeling technology is used to formally model the ideological and political course on the network platform, and the teaching process and learning process in the formal modeling are analyzed. Due to a large amount of data on the network platform and the sharing of information. In this paper, Petri net is established to model and analyze the shared dynamic data, which improves the problem of data redundancy in the teaching mode and improves the stability of the teaching platform. The results show that big data dynamic modeling technology can effectively improve the system model, optimize the feedback efficiency of the education system, and improve the applicability of the network platform application. Finally, explore the impact of network platforms on students' learning efficiency. Firstly, the data mobility in the education system is analyzed. With the growth of the liquidity index, the data changes nonlinearly. Therefore, we use dynamic modeling technology to analyze the changes in the number of students using network platforms. Compare the traditional teaching mode with the network teaching mode, and compare the ideological and political course with other courses. Through the analysis of discrete dynamic modeling, the experimental results show that the network teaching mode can improve the overall learning efficiency of students. In the learning process, preview and review are also the main factors affecting students' performance changes.

## Figures and Tables

**Figure 1:** Relationship between professor and learning system.

**Figure 2:** Comparison diagram of system stability before and after Petri net optimization.

**Figure 3:** Formal dynamic model of network teaching of ideological and political course under Petri net system.

**Figure 4:** Comparison of operation efficiency of network platform teaching system before and after Petri net optimization.

**Figure 5:** Comparison of operation speed between them in processing a large amount of data.

**Figure 6:** Trend chart of students' scores in various subjects.

**Figure 7:** Comparison between network platform teaching and traditional teaching. (a) Traditional teaching mode. (b) Network teaching mode.

**Figure 8:** Comparison chart of changes in learning ability.

**Figure 9:** Accuracy comparison between traditional modeling algorithm and big data dynamic modeling algorithm.

**Figure 10:** Comparison between prediction effect and actual effect.

## Data Availability

The figures used to support the findings of this study are included in the article.
